This article has been retracted.

# EV71 virus reduces Nrf2 activation to promote production of reactive oxygen species in infected cells

**DOI:** 10.1186/s13099-020-00361-w

**Published:** 2020-04-23

**Authors:** Zhenzi Bai, Xiaonan Zhao, Chenghua Li, Chuanlun Sheng, Hongyan Li

**Affiliations:** Infectious Department, China-Japan Union Hospital, Jilin University, No.126, Xiantai Street, Economic Development Zone, Changchun, 130033 Jilin China

**Keywords:** EV71 virus, Keap1, Nrf2, ROS, Apoptosis, Inflammation

## Abstract

**Background:**

Emerging evidence closely links Enterovirus 71 (EV71) infection with the generation of reactive oxygen species (ROS). Excess ROS results in apoptosis and exacerbates inflammatory reactions. The Keap1–Nrf2 axis serves as an essential oxidant counteracting pathway.

**Methods:**

The present study aimed to elucidate the role of the Keap1–Nrf2 pathway in modulating apoptosis and inflammatory reactions triggered by oxidative stress in Vero and RD cells upon EV71 infection.

**Results:**

Elevated ROS production was identified in EV71 infected Vero and RD cells. The percentage of dead cells and expression of inflammation-promoting cytokines were increased in these cells. EV71 infected cells also displayed reinforced Keap1 expression and abrogated Nrf2 expression. Keap1 silencing resulted in the downstream aggregation of the Nrf2 protein and heme oxygenase-1 HO-1. Keap1 silencing repressed ubiquitination and reinforced Nrf2 nuclear trafficking. Furthermore, silencing Keap1 expression repressed ROS production, cell death, and inflammatory reactions in EV71 infected RD and Vero cells. In contrast, silencing of both Keap1 and Nrf2 restored ROS production, cell death, and inflammatory reactions. Nrf2 and Keap1 modulated the stimulation of the Akt sensor and extrinsic as well as intrinsic cell death pathways, resulting in EV71-triggered cell death and inflammatory reactions.

**Conclusions:**

EV71 infection can trigger ROS production, cell death, and inflammatory reactions by modulating the Nrf2 and Keap1 levels of infected cells.

## Background

Hand, foot, and mouth disease (HFMD) is a viral infection that frequently occurs in infants and children. Common symptoms are blisters and flu-like symptoms [1–3]. HFMD is caused by several enteroviruses, including coxsackie virus A16 and enterovirus 71 (EV71) [4–6]. EV71 is a single positive RNA strand virus that belongs to the *Enterovirus* genus of the *Picornaviridae* family [7, 8]. EV71 infections are frequently linked to aggressive pulmonary, gastrointestinal, and neurological malfunctions in children. Additionally, the boosted generation and reaction of inflammation-promoting cytokines and chemokines influences the severity of EV71 infection [9].

Nuclear factor (erythroid-derived 2)-like 2 (Nrf2) and Kelch-like ECH-associated protein 1 (Keap1) have attracted attention concerning reactive oxygen species (ROS)-linked etiology. Expression of detoxifying enzymes (DEs) and antioxidant enzymes (AEs) is triggered by Nrf2, which is essential in the defense of vertebrates from stress in their surroundings [10]. Nrf2 can also enhance the activity of DE and AE related genes in protective responses to stresses that include ROS, reactive nitrogen species (RNS), and electrophiles [11, 12]. On the contrary, the dominant feature of Keap1 is as an oxidative stress (OS) sensor that specifically involves Nrf2, an E3 ubiquitin ligase substrate-recognizing subunit. Keap1 reinforces degeneration via the ubiquitin–proteasome system to repress Nrf2 in the absence of stress. The cysteine residue of Keap1 reduces Nrf2 ubiquitination in the presence of electrophiles or OS. The NRF2 protein triggers target expression via intracellular aggregation, which protects cells against surrounding stress.

ROS are crucial signaling agents that are essential for the development of inflammatory diseases [10]. Multiple downstream effects of reinforced OS (promotes ROS generation) are directly related to the stimulation of multiple inflammation cascades [11, 12]. The interaction between the inflammatory reactions and ROS has been recently investigated, with ROS arising from the mitochondria directly triggering agents that reinforce the expression of inflammatory cytokines via distinct pathways [13, 14]. Both ROS and mitochondria are crucial to stimulate cell death in physiologic and pathologic circumstances. ROS both arises from mitochondria and affects mitochondria. Cytochrome c generated from mitochondria stimulates caspases and seems to be dominantly regulated by ROS, either directly or indirectly [15]. ROS can modulate cell death at the transcription level by repressing the expression of viability-promoting proteins, including inhibitor of apoptosis proteins (IAPs), B cell lymphoma 2 (Bcl-2), survivin, and Bcl-XL, and reinforcing the expression of cell death-promoting agents [16]. ROS also stimulate the transcription of cell death-promoting genes that are critical in triggering intrinsic cell death pathways, including p53 upregulated modulator of apoptosis (Puma), Apoptotic protease activating factor 1 (Apaf-1), bcl-2-like protein 4 (Bax), Noxa, and BH3 interacting-domain death agonist (Bid), apart from extrinsic cell death-promoting agents, including Fas, Death receptor 4 (DR-4), Fas-L, and DR-5 [16]. The exact mechanisms of ROS-related inflammatory reactions and cell death in EV71 infection are unclear.

Our research explored the effect of EV71 infection on the stimulation and expression of Keap1–Nrf2 axis members using cell-based experiments. Furthermore, we elucidated the effect of Nrf2 and Keap1 on ROS production triggered by EV71 infection, and the effect of this ROS production on cell death, inflammation-promoting cytokine generation, and related signals. The findings revealed that the Keap1–Nrf2 axis is a crucial regulator of EV71-triggered ROS generation, inflammatory reactions, and cell death, with a crucial effect on viral replication.

## Materials and methods

### Cell cultivation

RD and Vero cells were provided by American Type Culture Collection and were cultured in Dulbecco’s modified Eagle’s medium (DMEM; Gibco) containing penicillin–streptomycin (2% v/v) and fetal bovine serum (FBS, 10%; Gibco) at 37 °C in an atmosphere of 5% CO_2_.

### Virus propagation

Human EV71 (GenBank accession number AF30299.1) stocks were produced in Vero cells, which were infected and then inoculated onto dishes (10 cm^2^). Vero cells were grown to near-80% confluency and were infected with EV71 virus diluted in DMEM. Aft a 1.5-h adsorption at 37 °C in a 5% CO_2_ atmosphere, the cells received DMEM containing 2% FBS. Infection continued until the monolayer demonstrated a cytopathic effect (CPE), 1 or 2 days after the infection. The cells and cultivation media were collected using a conical polypropylene tube and were treated using three freeze–thaw cycles. The final cell suspension was centrifuged for 10 min at 4500 rpm. The supernatant was removed, added to cryovials, and preserved at − 80 °C.

### TCID_50_ titration

The 50% tissue cultivating infectious dose (TCID_50_) titers were determined per ml. Briefly, Vero cells were seeded in 96-well plates (5 × 10^3^/well) 1 day prior to infection. DMEM containing 2% FBS (10^2^ to 10^7^) was utilized to serially dilute viruses, which were subsequently added to the wells. Plates were incubated from 2 to 5 days at 37 °C in a 5% CO_2_ atmosphere. The CPE was assessed by microscopy after the 2- to 5-day infection. The virus titer (TCID_50_) was examined by using the Reed–Muench endpoint calculation approach.

### EV71 infection

RD and Vero cells were infected with EV71 virus. Cell monolayers cultivated in 10 cm-diameter dishes to 50% confluency were treated with EV71 viruses at a multiplicity of infection (MOI) of 5 TCID_50_/cell. DMEM without FBS was used to wash the cells following a 1 h adsorption at 37 °C in a 5% CO_2_ atmosphere to eliminate virus that had not adhered. The cells then received fresh DMEM containing 10% FBS. The cells were sampled at defined times and analyzed.

### Small interfering RNA (siRNA) transfection

Cells were transiently treated with Keap1 siRNA and/or Nrf2 siRNA using Accell siRNA delivery medium (Dharmacon, USA) according to the manufacturer’s instructions. Cells (2 × 10^5^/well) were added to wells of 12-well plates and cultivated overnight at 37 °C in an atmosphere of 5% CO_2_. Then, 2 µm of Keap1 and Nrf2 siRNA (Smartpool, Dharmacon) in 1× siRNA buffer (Dharmacon) were transferred to each well, cultivated for 72 h at 37 °C and 5% CO_2_, and lysed. Keap1 and/or Nrf2 silencing efficiency was examined by qPCR.

### Western blotting

Cell lysates were collected using RIPA buffer. Proteins were resolved by 10% SDS-PAGE and transferred Immobilon polyvinylidene difluoride membranes with a pore size of 0.45 µm. Each membrane was blocked for 60 min using 5% bovine serum albumin at 25 °C. Primary antibody was added and incubated at 4 °C for 16 h, followed by the addition of secondary antibody for 1 h at 4 °C. Enhanced chemiluminescence was performed using the SuperSignal^®^ West Femto Maximum Sensitivity Substrate Kit (Thermo Fisher, Waltham, MA, USA) and a C-DiGit^®^ Blot Scanner (LiCor, USA).

### Quantitative real-time PCR (qPCR)

RNA was isolated from RD and Vero cells using TRIzol reagent (15596026, Invitrogen™). The transcription of various genes was quantified using SYBR Green master mix. Glyceraldehyde-3-phosphate dehydrogenase (GAPDH) served as the internal control. qPCR was carried out using a reaction volume of 0.02 mL in a RT-PCR system (Roche, Switzerland) and SYBR Green PCR master mix (Thermo Fisher Scientific). qPCR was conducted at 95 °C for 10 min, followed by 40 cycles of 60 °C for 15 s and 72 °C for 30 s. Copy number of the target genes was evaluated using the comparative CT approach (2^−ΔΔCT^) and an internal reference. The primer sequences are presented in Table 1.

**Table 1:** Sequences of primers

Primers	Sequences
VP1 F	5′-GCT CTA TAG GAG ATA GTG TGA GTA GGG-3′
VP1 R	5′-ATG ACT GCT CAC CTG CGT GTT-3′
Nrf2 F	5′-CTC GCT GGA AAA AGA AGT GG-3′
Nrf2 R	5′-CCG TCC AGG AGT TCA GAG AG-3′
Keap1 F	5′-TGG CCA GCG TGG AGT GCT AC-3′
Keap1 R	5′-TTG CAG CAA CAC CCG CTC CA-3′
IL-1β F	5′-TGA AAT GCC ACC TTT TGA CAG-3′
IL-1β R	5′-CCA CAG CCA CAA TGA GTG ATA C-3′
IL-6 F	5′-TGC CTT CTT GGG ACT GAT-3′
IL-6 R	5′-CTG GCT TTG TCT TTC TTG TT-3′
TNF-α F	5′-CGA TGA GGT CAA TCT GCC CA-3′
TNF-α R	5′-CCA GGT CAC TGT CCC AGC-3′
GAPDH F	5′-GGA AAG CTG TGG CGT GAT-3′
GAPDH R	5′-AAG GTG GAA GAA TGG GAG TT-3′

### Enzyme-linked immunosorbent assay (ELISA)

The supernatant was collected from the RD and Vero cells following the different treatments. The protein levels of interleukin-beta (IL-1β, BMS224; Invitrogen), IL-6 (BMS213, Invitrogen), and tumor necrosis factor-alpha (TNF-α, BMS622; Invitrogen) were determined using ELISA kits (Invitrogen™) following the manufacturer’s instructions. quantified using their corresponding standard curves.

### ROS production

ROS production in cells was examined using the 2ʹ,7ʹ-dichlorofluorescein diacetate (DCFH-DA) fluorescence probe. Subsequent to infection with EV71 for a defined time, the cells were incubated with DCFH-DA (10 µmol/L) for 0.5 h in the dark at 37 °C. Fluorescence intensity was assessed using excitation and emission wavelengths of 488 and 525 nm, respectively, using a model BX51 fluorescence microscope (Olympus, Japan).

### Terminal deoxynucleotidyl transferase dUTP nick end labeling (TUNEL) assay

The TUNEL fluorescence kit (Roche) was used for cell staining and assessment of cell death. 4′,6-Diamidino-2-phenylindole (DAPI, 1:5000; Beyotime, China) was used to stain the nuclei of cells. Cell death was assessed by calculating the number of TUNEL positive cells using a model SP8 laser scanning confocal microscope (Leica, Japan).

### Analysis of cell death

Cell death was assessed using Annexin V/propidium iodide (PI) staining and flow cytometry as previously described [17].

### Statistical analyses

Results are presented as average ± standard deviation (SD). Differences among the various groups were assessed using ANOVA and Tukey post hoc test. Differences among groups were assessed using the two-tailed t-test. A P-value < 0.05 was regarded as significant.

### Ethics statement

This study was approved by the Ethics Committee of China-Japan Union Hospital, Jilin University.

## Results

### EV71 infection stimulates ROS production, cell death, and inflammatory reaction of infected cells

RD and Vero cells were infected with EV71 virus at a MOI of 5. To assess the efficiency of infection, VP1 was found upregulated in both cells infected with EV71 at the mRNA and protein levels (Fig. 1a–c). Since ROS generation induces apoptosis and inflammation, we determined the ROS generation in EV-71 infected RD and Vero cells. EV71 infection resulted in remarkably increased ROS production in both cells (Fig. 1d). Next we determined the effect of EV71 infection on apoptosis and inflammation. Annexin V-FITC/PI flow cytometry revealed increased apoptosis in EV71 infected RD and Vero cells (Fig. 1e, f). Since excessive and robust pro-inflammatory cytokine production increases the severity of EV71 infection [10] and is highly relevant for apoptosis [20], production of these cytokines was investigated. The qPCR and ELISA data confirmed the significant increases in the levels of IL-1β, IL-6, and TNF-α mRNA and protein after EV71 infection (Fig. 1g, h).

**Fig. 1:** EV71 infection induces ROS generation, apoptosis, and inflammation of infected cells. **a**–**c** Reinforced mRNA and protein of VP1 in EV71-infected Vero and RD cells was identified in comparison to non-infected cells (Control) using western blotting and qPCR analyses. **d** ROS generation was examined in infected Vero and RD cells as evidenced by DCF fluorescence intensity assay compared to non-infected normal mice (Control). **e**, **f** Annexin V-FITC and PI flow cytometry was performed to assess the number of apoptotic Vero and RD cells. The upper right quadrant of every plot represents early dead cells. **g** qPCR analyses of the inflammation-promoting cytokines IL-1β, IL-6, and TNFα produced by infected cells. **h** The protein expression levels of IL-1β, IL-6, and TNFα of the infected cell were quantified using ELISA. Data are presented as mean ± SD. *P < 0.05, **P < 0.01, ***P < 0.001 vs. Control group

### EV71 infection mediates the Keap1–Nrf2 pathway

Since Keap1–Nrf2 axis played an essential role in the regulation of ROS production, we determined the expression level of Keap1 and Nrf2 in EV71-infected cells. Keap1 expression was reinforced in the infected cells, while the Nrf2 protein level was downregulated (Fig. 2a, b). qPCR was performed to assess the mRNA levels of Keap1 and Nrf2. The level of Keap1 mRNA was significantly increased in EV71-infected cells, while Nrf2 protein did not show any difference in the different groups (Fig. 2c, d). These data suggested that Nrf2 was regulated at the protein, rather than mRNA, level in the infected cells.

**Fig. 2:** EV71 infection upregulates Keap1 but downregulates Nrf2 levels. **a**, **b** Western blot to assess Keap1 and Nrf2 protein expression in the EV71-infected cells. **c**, **d** qPCR analysis to assess Keap1 and Nrf2 mRNA levels in the EV71-infected cells. Data are presented as mean ± SD. *P < 0.05, **P < 0.01 vs. Control group

### Silencing of Keap1 in EV71-infected cells influences downstream Nrf2 and HO-1 signals

To verify the effect of Keap1 on Nrf2 signal transduction during EV71 infection, Keap1 was silenced in Vero and RD cells prior to EV71 infection. Keap1 was downregulated upon transfection with Keap1 siRNA, whereas the downstream Nrf2 and HO-1 proteins were upregulated (Fig. 3a, b). EV71 infection resulted in the remarkable increase in Nrf2 ubiquitination, which contributed to Nrf2 reduction. In contrast, ubiquitination of Nrf2 was downregulated upon Keap1 depletion (Fig. 3c, d). Silencing of Keap1 significantly decreased Keap1 mRNA expression, while increasing HO-1 mRNA expression. However, Nrf2 mRNA expression was not altered (Fig. 3e–g). Since Nrf2 is mainly expressed in the nucleus, its subcellular localization was examined in each group using an immunofluorescence assay. EV71 infection resulted in the remarkable repression of Nrf2 nuclear translocation, but KEAP1 silencing in EV71 infected cells restored Nrf2 localization in the nucleus (Fig. 3h, i). These findings suggested that silencing of Keap1 influences the increased Nrf2 and HO-1 signaling in EV71-infected cells.

**Fig. 3:** Keap1 silencing upregulates Nrf2 activation in EV71-infected cells. Vero and RD cells were infected by EV71 at an MOI of 5 subsequent to 24 h transfection with Keap1 siRNA vector. **a**, **b** Western blot examination of the expression of Keap1, Nrf2, and HO-1 proteins in infected and non-infected cells. **c**, **d** Nrf2 was initially precipitated and western blot was performed to assess Nrf2 and ubiquitin. **e**–**g** qPCR was used to assess the mRNA of Keap1, Nrf2, and HO-1 in infected and non-infected cells. **h**, **i** Immunofluorescence was utilized to assess cytoplasmic as well as nuclear location of Nrf2 (tetramethylrhodamine, red). Nuclear DNA appears blue due to DAPI. Data are presented as mean ± SD. *P < 0.05, **P < 0.01 vs. Control group

### Silencing of Keap1 regulates ROS generation, apoptosis, and inflammation in EV71-infected cells

We further determined the effect of Keap1 silencing on ROS generation, apoptosis, and inflammation in EV71-infected cells. Excessive production of ROS following EV71 infection was significantly decreased after Keap1 silencing (Fig. 4a). Annexin V-fluorescein isothiocyanate and PI flow cytometry analyses showed that the apoptosis rate of infected Vero and RD cells was reduced due to KEAP1 downregulation (Fig. 4b, c). Findings of qPCR and ELISA suggested that Keap1 depletion substantially lessened the production of inflammation-promoting cytokines in EV71 infected RD and Vero cells at the mRNA and protein levels (Fig. 4d–i). The collective findings suggested that Keap1 modulates ROS production, apoptosis, and inflammation in EV71-infected RD and Vero cells.

**Fig. 4:** Keap1 silencing reduces ROS generation, apoptosis, and inflammation in EV71-infected cells. Vero and RD cells were infected by EV71 at an MOI of 5 subsequent to 24 h transfection using Keap1 siRNA vector. **a** DCF fluorescence intensity indicated ROS generation in the infected RD and Vero cells in comparison to non-infected normal mice (Control). **b**, **c** Quantity of dead RD as well as Vero cells using Annexin V-FITC and PI flow cytometry. The upper right quadrant of every plot stood for early dead cells. **d**–**f** Expression of inflammation-promoting cytokines IL-1β, IL-6, and TNF-α in the infected cells were assessed by qPCR. **g**–**i** The protein expression levels of IL-1β, IL-6, and TNF-α of the infected cells were quantified using ELISA. Data are presented as mean ± SD. *P < 0.05, **P < 0.01, ***P < 0.001 vs. Indicated group

### Nrf2 expression is responsible for Keap1-regulated, EV71-induced ROS generation

Keap1 and Nrf2 were co-silenced in EV71 infected cells to explore the effect of Nrf2 on ROS production, cell death, and inflammatory reactions. Nrf2 and downstream HO-1 expression were remarkably lessened at both the mRNA and protein levels subsequent to Nrf2 silencing, while Keap1 expression was unaffected even after Nrf2 silencing (Fig. 5a–e). These findings indicated that Nrf2 and Keap1 have appreciable effects on signaling pathways of RD and Vero cells infected with EV71. We then evaluated the effect of the co-silencing of Keap1 and Nrf2 on ROS production, apoptosis, and inflammation of EV71-infected RD and Vero cells. Nrf2 silencing recovered ROS production in cells, which was reduced by Keap1 depletion (Fig. 6a). Flow cytometry data indicated the Nrf2 silencing increased the proportion of apoptotic cells EV71-infected RD and Vero populations caused by Keap1-silencing (Fig. 6b, c). In addition, robust pro-inflammatory cytokine production was observed in the Keap1 and Nrf2 co-silencing group at both the mRNA and protein levels using qPCR and ELISA (Fig. 6d–i). These data demonstrated that Nrf2 is responsible for Keap1-mediated, EV71-induced cellular dysfunction. Because Akt phosphorylation is positively correlated with apoptosis and inflammation [18–20], we next assessed the effect of Nrf2 silencing on the activation of the Akt inflammatory sensor and the activity of proteins associated with cell death, including Caspase-3, Fas-L, Bax, and Fas. EV71 infection remarkably reinforced the expression of all these proteins (Fig. 7a, b), while depletion of Keap1 downregulated their expression. Notably, co-silencing of Nrf2 restored the cellular level of these proteins in the Keap1 silenced cells. These findings demonstrated that Keap1 can enhance EV71-triggered cell death and inflammation by reinforcing the concentrations of the cell death-promoting proteins and Akt phosphorylation, while Nrf2 downregulates them.

**Fig. 5:** Keap1 and Nrf2 co-silencing blocks Keap1–Nrf2–HO-1 transduction in EV71-infected cells. Subsequent to 24 h co-transfection with Keap1 and Nrf2 siRNA vectors, Vero and RD cells were infected by EV71 at an MOI of 5. **a**, **b** Western blot was used to examine the expression of Keap1, Nrf2, and HO-1 proteins in infected and non-infected cells. **c**–**e** qPCR was used to assess the mRNA of Keap1, Nrf2, and HO-1 in infected and non-infected cells. Data are presented as mean ± SD. *P < 0.05, **P < 0.01 vs. Indicated group

**Fig. 6:** Nrf2 silencing restores ROS generation, apoptosis, and inflammation of EV71-infected cells with Keap1 silencing. Subsequent to 24 h co-transfection with the Keap1 and Nrf2 siRNA vector, Vero and RD cells were infected by EV71 at an MOI of 5. **a** DCF fluorescence intensity indicated ROS generation in infected RD and Vero cells in comparison to the non-infected normal mice (Control). **b**, **c** Dead RD and Vero cells were enumerated using Annexin V-FITC and PI flow cytometry. The upper right quadrant of every plot stood for early dead cells. **d**–**f** Expression of inflammation-promoting cytokines IL-1β, IL-6, and TNFα in the infected cells were assessed using qPCR. **g**–**i** The protein expression levels of IL-1β, IL-6, and TNF-α of the infected cell were quantified using ELISA. Data are presented as mean ± SD. *P < 0.05, **P < 0.01, ***P < 0.001 vs. Indicated group

**Fig. 7:** Influence of Keap1 and Nrf2 on Akt activation and expression of pro-apoptotic proteins in EV71 infected cells. Subsequent to 24 h transfection using Keap1 and Nrf2 siRNA vector, Vero and RD cells were infected by EV71 at an MOI of 5. **a**, **b** Western blot demonstrated that Keap1 and Nrf2 silencing modulates Akt, phosphor Akt, Bax, Fas, Fas-L, Caspase-3, and cleaved Caspase-3 expression levels in EV71 infected Vero and RD cells

### EV71 propagation is regulated by Keap1 and Nrf2

Based on the above observations, we hypothesized that EV71 replication is regulated by Keap1 and Nrf2 silencing. To explore this, we assessed the virus replication rate in infected cells after Keap1 and/or Nrf2 silencing. Silencing of Keap1 reduced viral replication in RD and Vero cells, whereas Nrf2 silencing and co-silencing restored the virus titer 12 to 72 h post-infection (Fig. 8a, b). These results suggested that Nrf2 downregulation is required for efficient EV71 propagation.

**Fig. 8:** Effect of Keap1 and Nrf2 on EV71 replication. Vero and RD cells were initially transfected with Keap1 siRNA and/or Nrf2 siRNA, prior to infection with EV71 virus at an MOI of 5. **a**, **b** At defined times, viral titers were determined in the culture supernatants. Data are presented as mean ± SD

### Effect of ROS on EV71-induced apoptosis and inflammation

The effect of ROS has been demonstrated by treatment of EV71-infected cells with 10 μM of the ROS inhibitor *N*-acetyl-l-cysteine (NAC). Determinations of apoptosis and inflammation showed that NAC treatment contributed to a reductions in the number of EV71-induced apoptotic cells (Fig. 9a) and production of inflammatory factors (Fig. 9b), suggesting that ROS promoted the EV71-induced apoptosis and inflammation.

**Fig. 9:** Effect of ROS on EV71-triggered apoptosis and inflammation. Vero and RD cells were initially infected with EV71 virus at an MOI of 5 and then treated with 10 μM of the ROS inhibitor NAC for 5 h. **a** Quantity of dead RD and Vero cells were evaluated using Annexin V-FITC and PI flow cytometry. The upper right quadrant of every plot displays early dead cells. **b** The protein expression levels of IL-1β, IL-6, and TNF-α of the infected cell were quantified using ELISA. Data are presented as mean ± SD

## Discussion

Our data showed that EV71 infection triggered ROS generation, apoptosis, and inflammation of infected cells, and upregulated the expression of Keap1 but reduced the level of Nrf2. The induced ROS, apoptosis, and inflammation in the infected cells were decreased by Keap1 silencing but were restored by co-silencing of Keap1 and Nrf2 in Vero and RD cells. Additionally, reduced viral replication was observed after Keap1 silencing, while virus propagation was recovered by Nrf2 silencing. These findings strongly suggest that Keap1–Nrf2 axis exerts its regulatory effect on EV71 replication by inducing ROS production, apoptosis, and inflammation.

Redox homeostasis is an essential host factor contributing to the prognosis of infectious diseases. ROS generation is triggered by EV71 infection, which in turn reinforces viral replication [21]. Knowledge of the mechanism of EV71-triggered ROS generation is insufficient. Multiple viral and mitochondrial proteins influence one another, and can induce mitochondrial malfunction as well as the production of ROS. For instance, hepatitis B virus X protein (HBx, a hepatitis B viral protein) has an effect on mitochondrial heat shock proteins 60 and 70, and on voltage dependent anion channel 3 [22, 23], and triggers OS [24]. The core protein of HCV binds to mitochondria and reinforces OS [25–27]. The PB1-F2 protein of Influenza A virus targets mitochondria and induces abnormalities [28, 29]. EV71 infection reportedly triggers mitochondrial ROS production, which is crucial to viral replication and the consequent reduced efficiency of energy generation; the biogenesis of mitochondria is enhanced in infected cells to make up for the infection-related malfunction [30]. EV71 infection also increases ROS production [21, 30]. Nonetheless, the mechanism underlying ROS generation in cells infected by EV71 remains elusive, as is the ROS involved in the infection. Our research revealed that EV71 infection leads to a robust production of ROS, which may be involved in enhanced cellular apoptosis and viral replication. Administration of NAC ameliorated the apoptosis and inflammation of Vero and RD cells induced by EV71 infection. A plausible hypothesis is that apoptosis induced by ROS generation weakens the cellular membrane and facilitates the release of the viral particles. However, we did not identify the type of ROS involved in the EV71-mediated apoptosis and inflammation in Vero and RD cells, due to the non-specific nature of the DCFH-DA assay and the ROS scavenger NAC. The identification of ROS species during EV71-infected Vero and RD cells will be investigated in a future study.

Several studies have demonstrated the anti-oxidation and anti-inflammation effects of Nrf2 activation, and the generation of ROS during endogenous or exogenous cell oxidation stress. Nrf2 is dominantly bound to and is ubiquitinated by Keap1. Nrf2 localizes in the cytoplasm under physiological conditions. Nevertheless, Nrf2 can be translocated to the nucleus and can react with antioxidant agents, triggering the transcription of cytoprotective genes in response to electrophiles and OS. A majority of viruses bring about OS and reinforce the activities of radicals as well as ROS. These events cause the cellular immune system to stimulate Nrf2 and upregulate cytoprotective genes [31]. For instance, HO-1 is downregulated in the replication process of the Zika virus by regulating Nrf2 transcription factor expression or activity [32]. HBV [33], HCV [34], Dengue virus [35], Human immunodeficiency virus [36], Respiratory syncytial virus [37], and Marburg virus [38] activate Nrf2 and then elicit expression of antioxidant response genes, including NQO1, GSPT2, and HO-1. In addition, although our data demonstrated that EV71 infection enhance keapl expression in RD and Vero cells. However, the mechanism, by which EV71 enhances the expression of Keapl expression, is not identified. This mechanism might be related to EV71 survival. As a limitation of the present study, relevant investigation will be carried out in future. The present findings that EV71 infection results in Keap1 upregulation and Nrf2 downregulation differs from these previous studies. The expression of the Nrf2 protein was reduced upon EV71 infection, which contributed to increased ROS generation, and subsequently facilitated virus propagation.

## Conclusions

Our data strongly support a critical role of Keap1–Nrf2 signaling in EV71 proliferation in infected Vero and RD cells. Whether Keap1 and Nrf2 directly affect EV71 proliferation through apoptotic pathways or other signaling pathways requires further investigation. In the future, we will perform in vivo experiments in Keap1 and Nrf2 knockdown/knockout murine models to better understand these mechanisms.

## Data Availability

The datasets used and/or analyzed during the current study are available from the corresponding author on reasonable request.

## Abbreviations

HFMD: The hand, foot, and mouth disease
EV71: Enterovirus 71
ROS: Reactive oxygen species
Nrf2: Nuclear factor (erythroid-derived 2)-like 2
Keap1: Kelch-like ECH-associated protein 1
DEs: Expression of detoxifying enzymes
AEs: Antioxidant enzymes
RNS: Reactive nitrogen species
OS: Oxidative stress
MOI: Multiplicity of infection
FC: Flow cytometry
SD: Standard deviation
